The article "Full Endoscopic Surgery for Thoracic Pathology: Next Step after Mastering Lumbar and Cervical Endoscopic Spine Surgery?" was published in 2022. Journal: Biomed Res Int.

# Full Endoscopic Surgery for Thoracic Pathology: Next Step after Mastering Lumbar and Cervical Endoscopic Spine Surgery?

**DOI:** 10.1155/2022/8345736

**Published:** 2022-05-16

**Authors:** Junseok Bae, Sang-Ho Lee, Ralf Wagner, Jian Shen, Albert E. Telfeian

**Affiliations:** ^1^Wooridul Spine Hospital, Seoul, Republic of Korea; ^2^Ligamenta Spine Center, Frankfurt am Main, Germany; ^3^enVISION Spine Surgery, New York, NY, USA; ^4^Department of Neurosurgery, Rhode Island Hospital, The Warren Alpert Medical School of Brown University, Providence, RI, USA

## Abstract

Thoracic disc herniation and stenosis are relatively rare, and various symptoms make them difficult to diagnose. Due to the complexity of neural and vascular structure, surgical treatment of thoracic pathology is challenging. Endoscopic spine surgery is an emerging minimally invasive surgical option. Based on wide experience on the cervical and lumbar spine, an endoscopic approach for the thoracic pathology can be performed beyond the learning curve. Transforaminal approach for thoracic disc herniation, endoscopic unilateral approach, and bilateral decompression for thoracic stenosis have been reported as favorable and safe surgical options. In the present study, the authors described the detailed surgical procedure as well as tips and tricks.

## 1. Introduction

Thoracic disc herniation or thoracic stenosis is not common but causes axial back pain, radiculopathy, and myelopathy [1–6]. Traditional surgical approaches vary from laminectomy, transpedicular, transfacetal approach, lateral extracavitary approach, costotransversectomy, or transthoracic. These approaches have been performed successfully, but approach-related complications are inevitable. Especially, it is very important to identify the entry level of the magna radicular artery and avoid ligating it to prevent paraplegia caused by spinal cord infarction [7]. Overall, complications from open surgery are reported to occur in over 25% of patients [3].

Full endoscopic spine surgery is performed through a working-channel endoscope. The basic concept for the transforaminal or interlaminar approach is similar to the lumbar spine [8–10]. Endoscopic approaches to the thoracic spine have been reported and found to be safe and effective as well as avoiding approach-related complications with injury to the visceral and vascular structure [1, 2, 11–13].

In the present report, we review transforaminal endoscopic thoracic discectomy (TETD) and thoracic endoscopic unilateral laminectomy and bilateral decompression (TE-ULBD).

## 2. Material and Methods

### 2.1. Transforaminal Endoscopic Thoracic Discectomy

#### 2.1.1. Indication

Symptomatic soft disc herniation of paramedian, foraminal, or central disc space, not responding to the conservative treatment, is indicated for TETD. Symptoms can be varied from axial pain, radiculopathy, or myelopathy. Indications are important for beginners. Paramedian soft herniation with pain is the best indication for them. With experienced hands, challenging cases like myelopathy or calcified disc can be safely performed [1, 2, 11–13]. Concomitant ossification of the posterior longitudinal ligament or spinal infection is excluded.

#### 2.1.2. Surgical Instrument

Although the basic mechanics of instruments for the thoracic transforaminal endoscopy system is very similar to the lumbar endoscopy system, the subtle variations in angles, diameters, and length of instruments hold the key to the successful execution of thoracic endoscopic surgery.

(1) Thoracic endoscopes differ from other spinal endoscopes in the following ways (Figure 1):
  - They are angled at 45°. This allows to work with a steeper access route and much shorter in length as the thoracic spine does not have much soft tissue cover dorsally [2, 3, 12]
  - They are smaller in diameter to accommodate space restriction in the thoracic spine
(2) Endoreamers/endodrills are available in various sizes and angles. They are used for undercutting the superior facet or removal of a part of the vertebral body. They can also be used to make a hole in the annulus and allow easy passage of the dilator. They can also be used for the removal of small osteophytes or calcified disk material
(3) Instruments for discectomy are endoscopic forceps and dissecting instruments. There are rigid or articulating forceps either up biting or down biting figures. The jaws can be serrated or nonserrated. Radiofrequency probes can be used as a dissector and coagulator of soft tissue

#### 2.1.3. Procedures

The patient is placed in prone, and all procedure is performed under local anesthesia with conscious sedation.

An appropriate skin entry point was determined by drawing a line from the posterior annulus at the midpedicular level to the lateral margin of facet join on axial CT scans or MRI cuts (Figure 2). The skin entry point was commonly located at 5-6 cm from the midline. An oblique corridor is preferred, and the approach angle is measured by drawing a line on a lateral fluoroscopic view from the posterior endplate of the lower vertebra passing the tip of the superior articular process along with its inclination.

After infiltration of local anesthetics, an 18-gauge needle is advanced along the planned trajectory under lateral fluoroscopic view to the lateral aspect of the superior facet. A guidewire was inserted through the needle. Foraminoplasty was performed using sequential reamers. Alternative foraminoplasty techniques are (1) drilling the ventral aspect of the superior facet using a high-speed drill (Joimax® Shrill, 3.5 mm diamond burr) under direct endoscopic visualization and (2) using a Jamshidi needle to pass through the superior articular facet to reach at the midpedicular level on AP fluoroscopic view. A guidewire was inserted through the needle followed by serial dilation with side cutting bone drill inserted over the wire [3, 8, 14, 15] (Figure 3).

Epidurography was performed followed by an epidural block. Discography was performed by injecting a mixture of radiopaque dye and indigo carmine. Indigo carmine stains the degenerated acidic nucleus blue and helps in identifying the herniated disc fragment.

A beveled 5.8 mm outer diameter working cannula was then placed on the posterior disc space (Figure 4). Then, the 3.1 mm endoscope (TESSYS Thx, Joimax GmbH, Germany) was introduced. Under the direct visualization, a blue-stained annular surface and herniated disc fragment could be identified. By removing the annulus of the outer layer and the internal layer of the posterior longitudinal ligament (PLL) with a side-firing laser, the blue-stained herniated fragment was released from anchoring. Then, the fragment was removed using microforceps. After adequate decompression, ventral epidural space and thecal sac were visible. Epidural pulsation can be observed (Figure 5).

Resection of calcified disc herniation is composed of (1) epidural dissection between ventral dura and calcified disc, (2) cutting the annulus along the upper and lower endplate with endoscopic scissors or drilling the traction spur with articulating endoscopic burr, and (3) removal of a calcified disc with endoscopic forceps. Special attention is required to avoid dural injury in case of severe epidural adhesion [16, 17] (Figure 6).

The authors use a side-firing laser for TETD. Holmium:yttrium-aluminum-garnet (Ho: YAG) laser (VersaPulse; Lumenis, Yokneam, Israel) was used to ablate the posterior annulus and the PLL with minimal thermal necrosis. Ho: YAG laser is effective for (1) internal decompression within the posterior annulus at the initial stage, (2) shrinkage and resecting of the thickened posterior annulus around the annulus tear, (3) resecting of the PLL for exposing ventral epidural space for removal of transligamentous extrusion, and (4) resection of osteophyte or traction spur [2, 11, 17, 18].

### 2.2. Thoracic Endoscopic Unilateral Laminectomy and Bilateral Decompression

#### 2.2.1. Indication

The indication of TE-ULBD is single- or two-level thoracic spinal canal stenosis and ossification of the ligamentum flavum. Revision surgery and dural ossification are not recommended due to epidural adhesion and the risk of a dural leak. Lateral or extended type of OLF without no coexisting ossification of the posterior longitudinal ligament (OPLL) is best indicated for TE-ULBD.

#### 2.2.2. Surgical Instrument

A 7.3 mm outer diameter endoscope (iLESSYS Delta, Joimax GmbH, Germany) is used for the procedure. High-speed drill and endoscopic Kerrison rongeur are used for the decompression.

#### 2.2.3. Procedures

The patient is positioned prone under general anesthesia with neuromonitoring. A 1 cm skin incision is made on 1 cm lateral to the midline. Under the fluoroscopic guidance, serial dilators and a 10 mm working cannular are placed on the spinolaminar junction. A radiofrequency probe was used to clean soft tissue on the laminar. Unilateral laminectomy and subspinous process laminectomy are performed with a high-speed drill. An endoscopic Kerrison is used for resection of the ligamentum flavum. After exposing the upper and lower margin of ligamentum flavum, 1-2 mm of facet joint lateral to the dural sac needs to be drilled. With this technique, the OLF mass can be isolated for safe resection. In case of severe epidural adhesion, floating decompression can be considered than total resection to avoid dural tear. The floated mass should be very thin and soft for adequate dural decompression. It is important in floating decompression to make the OLF mass as thin as possible to make it light, then cut the margin to make it floating, and then try detaching it.

Bilateral decompression can be achieved by “over-the-top” decompression where the endoscopic drill is used for contralateral laminectomy via the subspinous process corridor [19]. Contralateral ligamentum flavum remains until bony decompression is achieved with the drill. The decompression is complete when the bilateral ligamentum flavum or OLF is removed and the dural pulsation is seen (Figure 7).

## 3. Discussion

Thoracic disc herniation and stenosis are relatively rare, and various symptoms make them difficult to diagnose. Due to the complexity of neural and vascular structure, surgical treatment of degenerative thoracic pathology is challenging [3, 14, 20–23]. Transforaminal approach offers the advantages of unique access to the spinal canal with minimal trauma of the anatomical structures, which make it superior to other surgical approaches for treating patients with chronic pain. In addition, there is little traction on the nerve, which can reduce nerve edema, and it does not cause excessive nerve tissue exposure, thus minimizing postoperative neural adhesion.

There are some steps requiring successful thoracic endoscopic surgery. Extensive experience for lumbar transforaminal approach, with wide range of foraminoplastic technique using various endoscopic instruments such as high-speed burr, reamers, hand drills, and spinal lasers, are mandatory for TETD. It is also important to understand the anatomical properties of the thoracic spine. For TE-ULBD, proficient experience for lumbar and cervical interlaminar decompression for unilateral approach and bilateral decompression is necessary for safe and successful outcomes.

There is little risk but a special caution is needed to prevent the damage of the Adamkiewicz artery, which is an important medullary artery, primarily located on the left side and is mostly branched between T9 and T11. When the segmental arteries are bifurcated from the intervertebral foramen to the radiculomedullary and intercostal branches, it is close to the lower portion of pedicle. Care should be taken not to damage this part with reamer while doing foraminoplasty.

For the TETD, understanding the neural foramen anatomy is important in surgical planning. The height of the neural foramen is smaller, and the extraforaminal space becomes narrower by the costovertebral joint, and the width of the foramen becomes wider because of the coronal oriented facet joint. From T1 to T10, The intervertebral foramen in the thoracic spine is characterized by the head of the closet rib, superior articular process and ventral aspect of facet joint, pedicle, ligamentous and capsular attachment, and the intervertebral disc. Extensive foraminoplasty is mandatory for the TETD in treating upper and middle thoracic level [1]. Neural foramen in the T10-11 and T11-12 level is similar with the upper lumbar spine because the 11th and 12th rib do not play a role in the structure. In this regard, it is recommend to start TETD from lower thoracic level after proficiency of lumbar endoscopic surgery [15].

It is important to differentiate dural ossification for TE-ULBD. There are two radiological signs of dural ossification, known as “tram-track or double-layer sign” and “comma-sign” [24]. The “tram-track sign” is characterized by a linear hyperdense bony excrescence with a central hypodensity. “Comma sign” is the ossification on half of the circumference of the dura mater. There is high risk of dural leak for those cases. Considering the technical limitations for dural repair by full-endoscopic approach, preoperative radiological review is important in selecting proper indications.

A recent systemic review of full endoscopic surgery for thoracic pathology showed international adaptation of endoscopy for thoracic disc herniation and stenosis with excellent outcomes and fewer complications than after open surgery. Excellent or good outcomes were achieved for full endoscopic procedures in a mean of 81% of patients (range 46–100%) with a complication rate of 8% (range 0–15%) [3].

In addition to the step-by-step surgical approach described above, there are some points to consider for the success and safety of endoscopic procedures.

1. Neuromonitoring: under general anesthesia, neuromonitoring including MEP and SSEP is essential. However, local anesthesia under conscious sedation provides “self-neuromonitoring” by allowing patients to respond to stimuli
2. Calcification: preoperative CT scan should be checked to identify calcification. Up to 70% of thoracic herniated disks are reported to be calcified at presentation, and 5–10% of calcified discs are associated with an intradural extension. In case of severe epidural adhesion, calcified herniation carries a high risk of dural tear. Internal decompression or floating decompression should be considered as an alternative to total resection of calcified hernia
3. Giant herniation: thoracic disc herniation occupies >40% of the spinal canal diameter that is frequently associated with myelopathy, calcification, intradural extension, and worse functional outcomes than those with smaller herniation. Care should be taken to avoid spinal cord compression during the procedure
4. Recurrent herniation: a recent largest clinical series reported 2.1% (2/98 patients) of recurrent herniation. There is least epidural adhesion after TETD. Revision TETD can be performed safely [2]
5. Incomplete decompression: lack of visualization of the entire fragment is a common cause of incomplete decompression. The transligamentous hernia should be explored by resection of PLL to expose ventral dura mater. Otherwise, subligamentous decompression can leave the epidural fragment behind. Another common clinical scenario is related to central migrated hernia, where endoscopic visualization is restricted by limited endoscopic moving radius at the narrow neural foramen. Extensive foraminotomy/foraminoplasty is necessary for highly migrated central disc herniation [25]

## 4. Conclusion

Full endoscopic surgery is a safe and effective minimally invasive surgical option for thoracic pathology. Minimally invasive techniques have brought a paradigm shift in the management of cervical/lumbar spinal conditions, and similar techniques have been extrapolated to the thoracic region as well. With high-resolution visualization and a tissue-preserving surgical approach, endoscopic surgery enhances patient outcomes. One obstacle is the learning curve problem. With sufficient experience in cervical and lumbar spine endoscopic surgery, it will be possible to safely operate on the thoracic spine.

## Figures and Tables

**Figure 1:** Comparison of intraoperative view of 45-degree working angled thoracic endoscopy (a) and 15-degree lumbar endoscopy (b) used for TETD. Note endoscopic field of view (yellow) is wider with thoracic endoscopy.

**Figure 2:** The skin entry point was determined by drawing a line from the posterior annulus at the midpedicular level to the lateral margin of the facet joint on axial computed tomography scan or magnetic resonance imaging, usually located approximately 6-7 cm from the midline.

**Figure 3:** Special surgical instrument used for foraminoplasty: (a) manual bone drill, (b) manual bone reamer, and (c) endoscopic high-speed burr.

**Figure 4:** Fluoroscopic view of transforaminal working channel placement. Note that it is located on the medial pedicle line on the AP view and the posterior vertebral line on the lateral view.

**Figure 5:** Intraoperative photo showing (a) the posterior longitudinal ligament (arrow) and thickened posterior annulus and (b) full decompression of dural sac (∗).

**Figure 6:** Case presentation of a 49-year-old female, presented with thoracic back pain and gait disturbance for a 3-year duration. Preoperative sagittal (a) and axial (b and d) MRI and CT scan (c and e) showing calcified disc herniation compressing the spinal cord at the T7-8 and T8-9 levels. Transforaminal endoscopic discectomy under local anesthesia was done using a high-speed articulating burr to drill bone spur (g). Postoperative sagittal (f) and axial (h and i) MRI shows full decompression and the patient's pain and myelopathy were improved.

**Figure 7:** Intraoperative endoscopic view showing (a) working channel is placed on the spinolaminar junction. (b) After laminectomy high-speed drill, upper margin of ligamentum flavum is exposed. (c) The decompression is complete when the bilateral ligamentum flavum or OLF is removed and the dural pulsation is seen.

## Data Availability

No data were used to support this study.
